# Is Increasing Age Associated with Higher Rates of Intercostal Arteries Vulnerable to Laceration? A Point of Care Ultrasound Study

**DOI:** 10.3390/jcm11195788

**Published:** 2022-09-29

**Authors:** Gerard Salame, Elizabeth Wittrock, Hardik Patel, Brant Hafen, Ayal Levi, Tyler Millard

**Affiliations:** Saint Joseph Hospital, Denver, CO 80218, USA; ellizabeth.wittrock@imail.org (E.W.); hardik.patel@cuanschutz.edu (H.P.); brant.hafen@gmail.com (B.H.); levi.56@osumc.edu (A.L.); tyler.j.millard@kp.org (T.M.)

**Keywords:** thoracentesis, point of care ultrasound, intercostal artery laceration, pre-procedural planning

## Abstract

Ultrasound-guided pre-procedural planning decreases complications from bedside thoracentesis. Although rare, intercostal artery (ICA) laceration is a serious complication that occurs when vulnerable intercostal arteries (VICA) are no longer protected by the superior rib. We sought to determine if increasing patient age is associated with greater odds of encountering a VICA. Randomly selected in-patients underwent pre-procedural planning for a mock posterior bedside thoracentesis. ICAs were categorized as vulnerable if they were visible within the corresponding intercostal space (ICS). We recorded where the VICA entered and exited the ICS as well as its unshielded length. A total of 40 patients (20 male) were enrolled and 240 ICS (6 ICS per patient) were scanned. Within this cohort, 25% of patients were noted to have at least one VICA. We could not demonstrate any relationship between the patient’s age or location of the ICS, with the odds of encountering a VICA (odds ratio (OR) = 1.0, *p* = 0.76; OR = 0.85, *p* = 0.27, respectively). Given the haphazard nature of VICA distribution and poor outcomes associated with inadvertent laceration, we recommend that ICA screening at the site of needle insertion be routinely performed prior to thoracentesis.

## 1. Introduction

Thoracentesis is a common bedside procedure performed by a multitude of medical, radiological, and surgical specialties. It is estimated that 176,000 thoracenteses are performed each year in the United States [1]. Position statements by the Society of Hospital Medicine (SHM) [2] and British Thoracic Society [3] highlight the importance of point of care ultrasound (POCUS) guided pre-procedural planning for thoracentesis. In one study, POCUS conducted pre-procedural planning decreased the rate of pneumothorax from 18% to 3% [4], in another analysis it reduced the cost of in-patient care, when compared to a landmark only based approach [5]. A less frequent complication associated with thoracentesis is intercostal artery (ICA) laceration and secondary hemothorax, estimated to occur in 0.2–2% of thoracenteses [6,7]. Aberrant or vulnerable ICAs (VICA) sagging into the intercostal space are at increased risk of laceration which can lead to life-threatening hemorrhage requiring invasive therapies such as open thoracotomy or ICA embolization [6,8] with case series suggesting higher survival rates with the former intervention [references to be added pending reviewer #2 Comments] versus the latter where mortality can reach up to 30% [8]. There is no clear guidance as to which patients need to be screened for these VICAs prior to thoracentesis. Prior literature has shown an increase in ICA tortuosity with increasing age [9,10,11]. We theorize that age-related increase in ICA tortuosity will lead to an increase in the frequency of detectable VICAs in older patients.

## 2. Materials and Methods

The study was conducted at Saint Joseph hospital in Denver, Colorado, 400-bed academic community hospital patients from the general medicine and surgical wards were randomly selected to participate in the study. Randomization was accomplished by having investigators verbally consent patients sequentially on each medical and surgical unit prior to chart review. They each were trained by the POCUS director in the proper technique for bedside ultrasound guided spinal mapping. The three ICS above the diaphragmatic level were scanned looking for VICAs.

Patients were eligible if they were: able to maintain a seated position, to consent, and admitted to the general inpatient surgical or medical teams. Patients were divided into 4 age groups: 18–49, 50–59, 60–69 and ≥70 years old, representing groups 1 to 4, respectively. Patient enrollment was not contingent on any plans for invasive pleural procedures. The patient’s age, body-mass index (BMI) and sex were recorded. Each patient was given a subject identification. Patients were excluded from the study if they were unable to meet the inclusion criteria or if they had soft tissue infections or rib fractures over the planned scanning area, The Colorado Multiple Institutional Review Board reviewed and approved this study. No identifiable patient health information was recorded, and patients were verbally consented.

POCUS images were acquired by 5 internal medicine residents (two postgraduate year (PGY) 3 residents, one PGY2, and one PGY1 from the Saint Joseph Hospital internal medicine residency program and by the Director of POCUS Education for that program. Image acquisition included ultrasound-guided mapping of spinous process level and their corresponding ICS (see details below). Prior to patient enrollment, residents received a 30 min didactic focusing on ultrasound-guided spine mapping as well as ICA image acquisition and optimization. To ensure proper technique, each resident, under the supervision of the POCUS director, practiced the acquisition protocol on 3 randomly selected in-patients. ICAs were deemed vulnerable (VICA) if the vessels were seen in the ICS and assumed to be shielded if they could not be visualized.

To mimic a posterior thoracentesis approach patients were asked to sit up on the side of the bed while leaning on a hospital end table. Investigators first mapped the spine using the approach described by Soni et al. [12] Using the abdominal deep setting of the Butterfly IQ+ probe © the hyperechoic and serrated bone line of the sacrum was identified in its transverse plane. From here the probe was moved rostral until superficial hyperechoic spinous processes with posterior shadowing were identified in the center of the screen (see Figure 1: Spinal and Rib mapping). The spinous processes and their respective ICS were mapped from L5 to T7 (where the tip of the scapula lies, an anatomic landmark used frequently for thoracentesis). 

Once spinal mapping was completed, the course of the ribs extruding from each spinous level was then drawn from the vertebral body until the posterior axillary line, by sliding the probe laterally from the spine while keeping the hyperechoic rib line centered on the ultrasound screen. The ICS at which the diaphragm was visualized at the mid-clavicular line, corresponding to its most rostral point along the posterior chest wall at end-expiration, was identified and noted as ICSdi. To avoid theoretical diaphragmatic laceration, we determined the lowest possible site to safely access the pleural cavity was one ICS above this location (noted as ICSdi + 1).

After mapping the spine and ribs posteriorly, investigators scanned each ICS starting at the ICSdi + 1 and the two ICS above it (ICSdi + 2 & ICSdi + 3). The protocol described by Salamonsen et al. [13]. was used to acquire and optimize the ICA image. The high frequency carotid setting of the Butterfly IQ+ © ultrasound system was used along with the color flow Doppler. The probe was kept perpendicular to the chest wall with the marker in the rostral position. Starting at the spinous process the probe was moved laterally until the ICS was visible. The superior and inferior ribs were kept on either side of the ultrasound screen while concomitantly centering the ICS. To improve ICA detection with color flow Doppler the probe was tilted in a medio-lateral plane every 1–2 cm while sliding laterally. If a vessel was visually identified but lacked the confirmatory pulsation with color flow Doppler, pulse wave Doppler was used to identify arterial pulsation tracing. The maximal distance from the inferior border of the superior rib and the inferior border of the artery (CoA) was measured using calipers available on the ultrasound device, (see Figure 2: Ultrasound landmarks and measurements). When visualized VICAs were followed laterally along the rib space until they migrated beneath the border of the superior rib. This distance was recorded and referred to as the unshielded length of the vessel (UnL). The distance between the spine and beginning and end points of the unshielded course of the VICA were recorded (Spino-Arterial Insertion or SpAi and Spino-Arterial exit or SpAe, respectively). This process was repeated from the ICSdi + 1 to ICSdi + 3 for each hemithorax, for a total of 6 scanned ICS per patient. For each patient, the total number of visualized shielded and vulnerable ICA was recorded.

Based on evidence in the literature, needle insertion for thoracentesis should occur 6 cm lateral to the spine as the rate of unshielded ICA proximal to this area is high [9]. In addition, Salamonsen et al., [13] showed that, when compared to Computerized Tomography (CT), ultrasound was sensitive but lacked specificity (86% and 30%, respectively) in identifying VICAs. The low specificity was thought to be secondary to false positives related to the ability of ultrasound beams to make shielded vessels appear in the ICS when the probe is not perpendicular to the skin. To correct for this error, the authors considered VICAs located in the top 0.3 cm of the ICS as protected. This correction increased specificity of VICA detection to 97%. Based on these findings, we excluded VICAs that met the above criteria. We refer to the remaining 19 observations as the adjusted vulnerable ICA cohort which was used in our final analysis. (See Figure 3: Adjusted Cohort).

## 3. Statistical Analysis

All data was processed using Stata17© software version 17.0. Given the binary nature of the dependent variable (the presence or absence of VICA) we used a logistic regression model to calculate OR with 95% confidence intervals and used *p* < 0.05 as the cutoff for statistical significance. The complete model examined the relationship between the presence of VICA and patient sex, age, age group, and Body Mass Index (BMI) as well as the ICS level and hemithorax. All predictor variables were treated as categorical except for BMI and age. The resulting coefficients represent the effect of 1 unit of the predictor variable on the OR of detecting a VICA.

A subgroup analysis of all VICAs was then performed using a multivariate regression analysis to assess for any association between unshielded length, entry and exit points of the VICA and number of VICAs with regard to sex, BMI, ICS, and age.

For quality assurance, 20% of patients scanned by residents were rescanned by the POCUS director, after all marks were removed from the patient. An inter-rater reliability Cohen’s Kappa coefficient was calculated using this cohort.

## 4. Results

A total of 44 patients and 264 ICS were scanned from spine to posterior axillary line; 23 VICAs were detected. Based on the methodology described above we excluded 4 VICAs, from 4 different patients leaving 40 patients in the final adjusted cohort. (See Figure 3: Adjusted Cohort) Of those, 10 patients had a total of 19 VICAs present. This cohort included: 20 female and 20 male patients, 240 ICSs split evenly between left and right hemithoraces. There was no statistically significant difference in age (59.1 vs. 62.4, *p* = 0.28), BMI (28.4 vs. 28.42 kg/m^2^, *p* = 0.5) between the final shielded and vulnerable groups, respectively.

One-quarter (10/40) of patients had at least one aberrant ICA that was detected by ultrasound. The probability of encountering an unshielded ICA within any of the three ICS above the diaphragmatic level was 7.9% (19 VICAs distributed among 240 ICS). We found no association between the continuous variable age (95% CI [0.96–1.02]), categorical variable age group (95% CI [0.63–1.4]) or ICS (95% CI [0.64–1.13]) with the OR of detecting VICA (see Table 1 Results). On Average VICA were first visualized 8.1 cm (CI 95% [6.4–9.7]) from the spine and remained exposed for 3.96 cm (95% CI [1.94–5.97] cm) and disappeared at 12.1 cm (95% CI [10.1–14.1]) from the spine. The mean maximal distance of the inferior wall of the vessel to the inferior border of the superior rib was 0.69 cm (CI 95% [0.52–0.86])

## 5. Discussion

ICA laceration is a rare but potentially serious complication that occurs when a VICA is severed while performing a thoracentesis [8]. Bedawi et al. showed that ultrasound-based ICA identification changed the site of pleural intervention in 15.6% cases [14]. Prior studies have demonstrated increasing tortuosity of ICA with increasing patient age [10,15,16]. We sought to determine age related increase in tortuosity translated to higher rates of VICA detection.

To our knowledge, this is the first study evaluating the ICA position continuously across the posterior chest wall using POCUS. Prior studies used CT with special software to delineate the ICA path along this region [9,15] which is not routinely available or performed prior to thoracentesis. Our approach mimicked the ultrasound guided pre-procedural planning for bedside thoracentesis recommended by the SHM© [2] and BTS© [3] and allows for bedside assessment of ICA position.

We could not demonstrate an association between age and the frequency of VICA detection (see Table 1). Instead, our findings strengthen prior literature demonstrating a wide variability in ICA path regardless of age [9,11,17,18]. In addition, sex, ICS level and BMI had no statistically significant impact on the OR of detecting a VICA.

In our final cohort, 25% of our patients had at least one VICA along their posterior chest wall. The rate of ICA laceration reported is far lower and estimated at 0.2–2% [6,7]. This discrepancy is thought to be due to the small space that these aberrant vessels occupy relative to the total intercostal area.

In our subgroup analysis of the VICA cohort, the unshielded length of the aberrant vessels was similar to that seen in Helm et al. with a mean of 3.9 cm [9]. The average CoA depth in our cohort was 0.69 cm (CI 95% [0.52–0.86]), like that noted by Dewhurst et al. (CoA 0.56 ± 0.05 cm) [18]. Variation in the course of posterior ICA has already been extensively described [9,11,17] the only pattern that has been consistent throughout the literature is the tendency of the posterior ICA to migrate towards the superior rib as it moves more laterally across the chest wall [13,15,18]. This tendency has led multiple authors and the BTS© [3] to advocate for a more lateral approach when feasible for invasive pleural procedures. We noted a similar pattern in our study where on average for every centimeter lateral to the spine VICAs migrated almost 1 mm closer to its superior rib. In our cohort VICAs were visualized as far as 14.1 cm from the spine. This corresponds to the posterior midclavicular region in most patients, an area commonly used for pleural cavity access. CT studies have localized aberrant ICA as far as the posterior axillary line [13,15]

The haphazard nature of posterior ICA path makes it difficult to predict which patients will have VICA prone to laceration as well as the location of such vessels on the posterior chest wall. Identifying VICAs using bedside ultrasound can be done in less than one minute with high sensitivity and specificity [13]. These test characteristics make POCUS an appealing tool to potentially decrease the rate of VICA laceration, which has been associated with a 90-day mortality rate of 30.6% [8].

These findings must be tempered with our small sample size. Larger studies would be needed to increase the generalizability of our results and lead to a change in routine clinical practice.

## 6. Conclusions

Our study demonstrated that age was not associated with an increasing frequency of VICA. However, it did reveal that VICAs are more common than previously thought, something that clinicians may not be aware of. Our results could not detect any patient related variables to help guide patient selection for pre-procedural screening for VICAs. The unpredictable nature of VICAs in combination with the high rates of invasive intervention and mortality, associated with iatrogenic ICA laceration [8], and negligible time required for VICA identification by bedside POCUS [13], support including an evaluation for VICAs for all thoracenteses as a routine part of POCUS guided pre-procedural planning. Alternatively, choosing more lateral approaches where aberrant ICA are typically closer to the superior rib may decrease the rate of ICA laceration. Larger, multi-institutional studies are needed to assess the impact of pre-procedural VICA detection on rates of ICA laceration.

## Figures and Tables

**Figure 1:** Spinal and Rib mapping. (**a**) Schematic representation, (**b**) Measurements on patient’s back. Legend: Blue line depicts the diaphragm. ICSdi: refers to the ICS at mid-axillary line where the diaphragm was seen ICSdi + 1 to +3 refers to ICS level above the ICSdi and represent the scanned areas. Measurements were done using a paper ruler in cm, SpAi: (yellow arrow), distance between spinal column (Orange line) and initial entry of Intercostal artery into the intercostal space, SpAe: (Orange Arrow) distance between spinal column and exit of intercostal artery from the intercostal space, Green segment of intercostal artery represents its unshielded length (UnL), and is equal to SpAe—SpAi.

**Figure 2:** Ultrasound landmarks and measurements. (**a**) Schematic Representation, (**b**) Ultrasound View. Legend: Probe is oriented in a rostro-caudal plane with marker pointed towards the patient’s head. ICSL: Intercostal space length (green double arrow) represents the distance between the superior and inferior rib borders, ICA: Intercostal Artery, Costo-Arterial distance (CoA) represents the distance from the inferior border of the superior rib to the inferior border of the ICA (blue double arrow).

**Figure 3:** Adjusted Cohort. Legend: ICA: Intercostal Artery, VICA: Vulnerable ICA, CoA: Distance of the inferior border of the ICA to the inferior border of the superior rib, ICS: Intercostal Space. * VICAs were excluded if they were within 6 cm of the spine or located in the rostral 0.3 cm of the ICS. ** Adjusted Cohort was used in final data analysis.

**Table 1:** Odds Ratio of detecting Vulnerable Intercostal Arteries.

Variable	Coeff	*p* Value	95% CI
Age Group *	0.95	0.81	[0.63–1.4]
Age	1.0	0.76	[0.96–1.02]
BMI	1.1	0.03	[1.01–1.2]
Gender	0.12	0.57	[0.5–3.8]
ICS	0.85	0.27	[0.64–1.13]

Legend: Coefficients represent the change in the Odds Ratio of detecting a vulnerable intercostal artery (VICA) when all other variables are held constant. ICS: Intercostal Space; ICA: Intercostal Artery; OR: Odds Ratio; BMI: Basal Metabolic Index. Statistical significance was defined as a *p*-value of less than 0.05. * Age Group: Patients were divided into 4 groups 18–49, 50–59, 60–69 and ≥70 years of age.

## Data Availability

The data supporting our findings are available to the editors and their staff upon request by contacting the corresponding author. This includes de-identified data of patient characteristics and raw data of intercostal artery measurements.
